# Separation and confirmation of nine Enterobacteriaceae strains that carry the *bla*_NDM-1_ gene

**DOI:** 10.3892/etm.2015.2255

**Published:** 2015-02-03

**Authors:** TIAN-JIAO LI, CHEN-XUE LI, SHU-PING CHENG, XU-MING WANG, SHENG-MIAO FU, XIAO-JUAN LI, TAO HUANG, HUI-QUN FU, SONG LIN, YE LU

**Affiliations:** 1 Department of Medical Examination, Hainan Provincial People’s Hospital, Haikou, Hainan 570311, P.R. China; 2 College of Agriculture, Hainan University, Haikou, Hainan 570228, P.R. China; 3 Department of Laboratory, Hainan Provincial Agricultural Reclamation General Hospital, Haikou, Hainan 570311, P.R. China; 4 Department of Laboratory, Traditional Chinese Medicine Hospital of Hainan Province, Haikou, Hainan 570203, P.R. China

**Keywords:** carbapenem resistance, *bla*_NDM-1_ gene, Enterobacteriaceae, Hainan, China

## Abstract

The aim of the present study was to confirm the existence of carbapenem-resistant Enterobacteriaceae carrying the *bla*_NDM-1_ gene in clinics in Hainan province, China. Collected clinical bacterial isolates that were Enterobacteriaceae strains suspected of producing carbapenemase were used as experimental strains. Drug resistance to imipenem, meropenem and other antibacterial agents was tested. Imipenem/imipenem inhibitor (IP/IPI) E-testing was conducted to identify the bacterial strains that produced metallo-β-lactamases. The *bla*_NDM-1_ drug resistance gene was amplified by polymerase chain reaction (PCR), and agarose gel electrophoresis (AGE) and sequencing were conducted to identify the products. The species of the strains carrying the *bla*_NDM-1_ gene were determined using a biochemical identification system. Through the IP/IPI E-test, 21 of the 30 collected Enterobacteriaceae strains were found to be positive, indicating that 70% of the strains produced metallo-β-lactamases. Following *bla*_NDM-1_ gene PCR amplification, AGE and sequencing tests confirmed that nine of the strains carried the *bla*_NDM-1_ drug resistance gene. The biochemical identification system indicated that four of the strains were *Klebsiella pneumoniae*, two were *Escherichia coli*, two were *Enterobacter cloacae* and one was *Enterobacter aerogenes*. Drug susceptibility testing *in vitro* demonstrated that the strains were 100% resistant to a broad spectrum antibiotic plus lactamase inhibitor, cephalosporins and carbapenems. However, they had high sensitivity rates to polymyxin B and tigecycline of 100 and 88.9%, respectively. The sensitivity rate to amikacin was also high at 77.8%, whereas sensitivity to ciprofloxacin and gentamicin was moderate at rates of 44.4 and 33.3% respectively. This clinical study of Enterobacteriaceae strains that carry the *bla*_NDM-1_ gene in Hainan shows a bacterial tolerance that is different from that in previous studies, which requires further in-depth study.

## Introduction

The enzyme New Delhi metallo-β-lactamase-1 (NDM-1) is expressed by certain bacteria that carry the *bla*_NDM-1_ gene. The earliest report of NDM-1 was by Yong *et al* (1) in December 2009. Yong *et al* separated a strain of *Klebsiella pneumoniae* that exhibited resistance to antibacterial agents such as carbapenems from the urine specimen of an Indian patient who was suffering from urinary tract infection in Sweden, confirming that the resistance mechanism of *Klebsiella pneumoniae* had led to the production of a new metalloenzyme. As this patient had once received treatment in New Delhi, the enzyme was designated NDM-1. An article published in The Lancet Infectious Diseases in August 2010 (2) reported that there had been 37 cases of Enterobacteriaceae carrying the *bla*_NDM-1_ gene in England, 44 in Chennai, India, 26 in Haryana, India, and 73 in other parts of India and in Pakistan.

Since the NDM-1 drug resistance gene can reduce the antibacterial activity of almost all β-lactam antibiotics, including the most potent carbapenem antibiotics, its presence in bacteria results in serious bacterial resistance. Drug resistance genes can be transferred by plasmid; hence, these features of NDM-1 may cause global public health security issues. The initial article in The Lancet Infectious Diseases drew worldwide attention. Shortly thereafter, the United States, Canada, Sweden, Greece, Israel, the Netherlands, Japan, Brazil and other countries (3), as well as Hong Kong (4) and Taiwan (5) in China began to carry out research into *bla*_NDM-1_. The Chinese Ministry of Public Health also made an announcement on October 25, 2010, requiring all medical institutions to screen and monitor bacterial strains containing NDM-1. To date, very few studies concerning the NDM-1 drug resistance gene have been published.

In 2011, clinical observations of Enterobacteriaceae strains that had a sharp reduction of sensitivity to carbapenem antibiotics and were suspected of carrying the *bla*_NDM-1_ gene began in Hainan. The current study investigated the existence of the *bla*_NDM-1_ gene in 30 Enterobacteriaceae strains collected in Hainan, and determined the species of these strains.

## Materials and methods

### Materials

The patients in this study attended the Hainan Provincial Agricultural Reclamation General Hospital and Traditional Chinese Medicine Hospital of Hainan Province (both Haikou, China) from January to December in 2012. In total, 30 Enterobacteriaceae strains were isolated from the patients and following the use of broth enrichment, were preserved at −70°C. The present study was approved by the Medical Ethics Committee of Hainan General Hospital (Haikou, China). Informed consent was obtained from the patients or patients’ families prior to their involvement in the present study.

### Reagents and instruments

The API 20E biochemical identification system (bioMerieux, Inc., Marcy l’Étoile, France) was used to identify the bacteria. The VITEK2 automatic bacterial identification and antibiotic susceptibility testing system (bioMerieux, Inc.) with supporting reagents, and imipenem, meropenem, tigecycline susceptibility and imipenem/imipenem inhibitor (IP/IPI) E-test strips (AB Biodisk, bioMerieux Inc., Stockholm, Sweden) were used to evaluate drug sensitivity and identify the metallo-β-lactamase phenotype. An E-Cycle™ 96PCR cycler (CapitalBio Corporation, Beijing, China), agarose gel electrophoresis (AGE) apparatus (Beijing 61 Instrument Factory, Beijing, China), JS-380 automatic gel imaging system used in AGE (Peiqing Inc., Shanghai, China) and 2X Power Taq PCR Master Mix (PR1700; BioTeke Corporation, Beijing, China) kit were used in the polymerase chain reaction (PCR) amplification process and a D2000 DNA Marker (MD114; Tiangen Biotech Co., Ltd, Beijing, China) was used as an AGE marker.

### Strain identification and drug sensitivity test

The API 20E biochemical identification system was used to identify bacteria, using the specific methods described by the manufacturer. The concentration gradient-based E-test strip method was used to measure the minimum inhibitory concentration (MIC) values (Fig. 1) in imipenem and meropenem *in vitro* susceptibility tests; the 2010 Clinical Laboratory Standards Institute (CLSI) threshold (6) was used to judge the sensitivity, medium and drug resistance. The E-test strip method was also used to test *in vitro* susceptibility to tigecycline; the results were determined in accordance with the US Food and Drug Administration Enterobacteriaceae criteria (an MIC ≤2 μg/ml is defined as sensitive; Fig. 2) (7). The VITEK2 automated bacterial identification system and supporting reagents were used to determine susceptibility (MIC values) to other antibacterial agents; the 2010 CLSI threshold (6) was used to judge the sensitivity, medium and drug resistance.

### Confirmation of metallo-β-lactamase phenotype

IP/IPI E-test papers were used to test the target bacterial strains as follows: The strains were cultured overnight. Sterile saline was used to dilute the suspension to 0.5 McFarland turbidity. The bacteria were coated onto the Müller-Hinton (MH) agar plate, the plate was allowed to dry for 10 min, the IP/IPI E-test strip was placed on the surface of the agar plate, and the plate was incubated for 16–18 h at 35°C. An IP/IPI ratio >8 indicated a positive result (Fig. 3).

### Extraction of bacterial DNA

The fresh culture was put into 100–200 μl sterile deionized water, boiled for 10 min and then subjected to centrifugation at 14,800 × g for 5 min. The supernatant fluid was extracted and preserved at −20°C.

### PCR amplification and sequencing

In the screening for the NDM-1-encoding gene, the primer sequences used and the PCR product details are shown in Table I. The PCR reaction conditions were initial denaturation at 94°C for 5 min; degeneration at 94°C for 15 sec, annealing at 55°C for 30 sec and 72°C for 30 sec, for a total of 25 cycles; followed by extension at 72°C for 5 min. Following the PCR amplification, 1.5% AGE of the products was conducted at 120 V for 40 min and the JS-380 imaging system was used to observe the results and capture photographic images. The products were submitted to Shanghai Biological Engineering Co., Ltd. (Shanghai, China) to conduct the sequencing. For full-length *bla*_NDM-1_ gene detection, the primer was designed with reference to FN396876.1 in Genbank, with details as shown in Table I. The acquired sequences along with the nucleotide sequence of FN396876.1 were entered into DNAStar software (DNASTAR Inc., Madison, WI, USA) and sequence alignment was performed by the ClustalW method. The PCR reaction conditions and processing for the full-length gene were the same as those described for the screening PCR.

### Quality control strains

The quality control strain for bacterial identification and drug susceptibility testing was ATCC25922 *Escherichia coli*, acquired from the Clinical Inspection Center of the Ministry of Health (Beijing, China).

## Results

### Results of screening for metalloenzyme production

When the samples were analyzed using the IP/IPI E-test, 21 of the 30 collected Enterobacteriaceae strains were found to be positive, confirming that 70% of the bacterial strains were producing carbapenemases of the metallo-β-lactamase phenotype.

### Results of bla_NDM-1_ gene screening by PCR amplification and sequencing

It was found that nine of the 21 strains that produced metallo-β-lactamase also presented positive segments at 292 bp (Fig. 4). Through DNA sequencing and DNAStar analysis, compared with the FN396876.1 sequence in GenBank, the homology comparison result was 100% in each case (reverse, 2751–2993), confirming that nine of the strains carried the *bla*_NDM-1_ gene.

### Results of full-length bla_NDM-1_ gene screening by PCR amplification and sequencing

Nine Enterobacteriaceae strains were carriers of the NDM-1-encoding gene; following full-length *bla*_NDM-1_ gene amplification, all nine strains exhibited positive results with bands at 1,001 bp (Fig. 5). Through sequencing and DNASTAR analysis, compared with the FN396876.1 sequence in GenBank, the homology was 100%. The gene sequences of certain strains were registered in GenBank; the accession numbers were KC573881.1, KC573880.1 and KC573878.1.

### Results of strain identification and susceptibility tests

Following testing with the API 20E biochemical identification system, four strains were identified to be *Klebsiella pneumoniae* (Nos. 1, 5, 6 and 8), two strains were *Escherichia coli* (Nos. 4 and 9), two strains were *Enterobacter cloacae* (Nos. 2 and 3) and one strain was *Enterobacter aerogenes* (No. 7). Specific information concerning the types of bacteria and drug susceptibility results are shown in Table II. The sensitivity rate of the *bla*_NDM-1_-positive strains *in vitro* was 77.8% to amikacin, 44.4% to ciprofloxacin and 33.3% to gentamicin. The sensitivity rates to polymyxin and tigecycline were 100 and 88.9%, respectively.

## Discussion

Carbapenem antibiotics are atypical β-lactam antibiotics with a broad spectrum and strong antibacterial activity. In the past 20 years, along with the increasing clinical use of cephalosporins, the rate of multi-resistant bacteria that produce high levels of AmpC enzymes and extended-spectrum β-lactamases (ESBLs) has also increased sharply (8) Thus, carbapenems have been used to treat illness caused by drugs that induce the production of AmpC enzymes and ESBLs. However, with the worldwide use of carbapenems as antibacterial agents in AmpC- and ESBL-producing bacteria and other multi-drug resistant bacteria, carbapenem-resistant Enterobacteriaceae (CRE) such as *Pseudomonas aeruginosa* and *Acinetobacter* have become prevalent in the clinic (9). In recent years, the clinical treatment and control of CRE infection has faced great challenges. In 2009, guidelines for CRE infection control in hospitals were published (10). This indicates that CRE had already begun to attract worldwide attention. The resistance mechanism of CRE is mainly due to the production of carbapenemases (11–13).

Carbapenemases are β-lactamases that are able to hydrolyze carbapenem antibiotics, including those of the A, B and D types according to the Ambler molecular classification. Carbapenemases may be of metal-free or metal-containing types. The former type includes NmcA and SME-1, while the latter includes L1, IMP-1 and VIM-1. NDM-1 is a gene that encodes a class B carbapenemase which hydrolyzes and inactivates the overwhelming majority of carbapenem antibiotics. Unlike the L1, IMP-1 and VIM-1 metallo-β-lactamase genes, the *bla*_NDM-1_ gene is located on a 140-kb plasmid (2), which can be transferred at a horizontal level between bacteria. It has been confirmed that strains with the *bla*_NDM-1_ gene can lead to the emergence and spread of multi-resistant bacteria among different species of bacteria (14). Hence, it is suggested that the monitoring and research of strains carrying the *bla*_NDM-1_ gene may be useful in preventing and controlling new types of multi-resistant bacteria.

Among the nine *bla*_NDM-1_-expressing Enterobacteriaceae samples isolated from various parts of the body of different patients in the present study, five were isolated from sputum, two were separated from the blood, and the other two were isolated from urine. The older patients had underlying diseases, including chronic obstructive pulmonary disease, cerebral infarction, hypertension and coronary heart disease, and had no medical history from other provinces or countries. Four patients were in an intensive care unit while the other five were from intensive medicine and geriatric, neurology, neurosurgery and endocrinology departments, respectively. Considering the history of the patients, it appears that the nine strains were local bacteria.

At present, there are very few reports from China concerning bacteria carrying the *bla*_NDM-1_ gene, and even fewer on Enterobacteriaceae carrying *bla*_NDM-1_. On October 26, 2010, the Chinese Military Academy of Medical Sciences and the Chinese Center for Disease Control and Prevention announced that three strains carrying the *bla*_NDM-1_ gene had been found in mainland China, two of which were enterococci from the feces of infants with diarrhea from Ningxia province (15) and the third was *Acinetobacter baumannii* in a sputum specimen from a lung cancer patient in Fujian province (16). A study reported in August 2011 that the gene had been identified in three strains of *Acinetobacter* and a case of *Klebsiella ozaenae* in Guangzhou (17). A strain of a *Klebsiella oxytoca* carrying the gene in Yunnan was reported in 2012 (18). A study from Hunan published in August 2012 reported that *Klebsiella pneumoniae* carrying *bla*_NDM-1_ had been isolated from the sputum specimen of a 8-month-old infant (19). In comparison with these other provinces, Hainan has a greater quantity of the *bla*_NDM-1_-carrying bacteria, which are from different bacterial genera. Among these bacteria, four are *Klebsiella pneumoniae*, two are *Escherichia coli*, two are *Enterobacter cloacae* and one is *Enterobacter aerogenes*.

The sensitivity rate of the *bla*_NDM-1_-positive strains *in vitro* was 77.8% to amikacin, 44.4% to ciprofloxacin and 33.3% to gentamicin. The strains were highly sensitive to amikacin but only moderately sensitive to ciprofloxacin and gentamicin. In a previous study by Kumarasamy *et al* (2), the sensitivity rates of 180 NDM-1-producing Enterobacteriaceae strains to gentamicin and ciprofloxacin were only 5–10%. The sensitivity rates to polymyxin (100%) and tigecycline (88.9%) in the present study are similar to those in the study by Kumarasamy *et al* (2), which were 80–90 and 90%, respectively. Resistance to broad-spectrum antibiotic plus β-lactamase inhibitor, cephalosporins and carbapenems has reached 100%, which is in agreement with the study by Kumarasamy *et al* (2).

Therefore, it appears that the isolated Enterobacteriaceae strains carrying the *bla*_NDM-1_ gene have different biological behaviors, which requires further in-depth study.

## Figures and Tables

**Figure 1:** Imipenem and meropenem E-test method result. Minimum inhibitory concentration, >32 μg/ml.

**Figure 2:** Tigecycline E-test method result. Minimum inhibitory concentration, 0.38 μg/ml.

**Figure 3:** IP/IPI E-test test strip results. IP/IPI >8 is considered MBL-positive. IP, imipenem; IPI, imipenem inhibitor; MBL, metallo-β-lactamase.

**Figure 4:** Electrophoresis results for the PCR products of nine strains of NDM-1-positive resistant gene (DNA fragment at 287bp). Lane M, marker (D2000); Lane B, blank control; Lanes 1, 5, 6 and 8, pulmonary bacteria; Lanes 4 and 9, bacteria from the large intestine; Lanes 2 and 3, *Enterobacter cloacae*; Lane 7, *Enterobacter aerogenes*. Lanes 1–9 show NDM-1 positive strains. NMD-1, New Delhi metallo-β-lactamase-1.

**Figure 5:** Electrophoresis results for the full-length PCR products of nine strains carrying the *bla*_NDM-1_ resistance gene (DNA fragment, 1,001 bp). Lane M, marker (D2000); lanes 1, 5, 6 and 8, *Klebsiella pneumoniae*; lanes 4 and 9, *Escherichia coli*; lanes 2 and 3, *Enterobacter cloacae*; lane 7, *Enterobacter aerogenes*; lane B, blank control.

**Table I:** PCR primers.

Primer	Details	Primer sequences (5′-3′)	Product length (bp)	Amplified fragment, location of CDS
Screening	Forward	CAGCACACTTCCTATCTC	292	Reverse, 2751–2993
	Reverse	CCGCAACCATCCCCTCTT		
Full-length	Upstream	TCGCATAAAACGCCTCTG	1001	Forward, 2564–3444
	Downstream	GAAACTGTCGCACCTCAT		

PCR, polymerase chain reaction; CDS, coding sequence.

**Table II:** Bacterial susceptibility results (μg/ml).

Variable	Bacterial strain no.									Sensitivity rate (%)

	1	2	3	4	5	6	7	8	9	
Strain type	*Kpn*	*Ecl*	*Ecl*	*Eco*	*Kpn*	*Kpn*	*Eae*	*Kpn*	*Ec*o	
Antibacterial agent										
Polymyxin B	≤2	≤2	≤2	≤2	≤2	≤2	≤2	≤2	≤2	100
Tigecycline (E-test strip)	1	0.75	1	1.5	3	1	1	1	0.25	88.9
Amikacin	8	≥64	≥64	8	8	8	≤2	≤2	≤2	77.8
Ciprofloxacin	≤0.25	≥4	≥4	≥4	≤0.25	≤0.25	≤0.25	2	≥4	44.4
Gentamicin	≥16	≥16	≥16	≤1	≤1	≥16	≤1	≥16	≥16	33.3
Cotrimoxazole	≥320	≥320	≥320	≥320	≤20	≥320	≥320	≥320	≥320	11.1
Aztreonam	≥64	≥64	≥64	≥64	≥64	≥64	≥64	≥64	16	0
Ceftazidime	≥64	≥64	≥64	≥64	≥64	≥64	≥64	≥64	≥64	0
Ceftriaxone	≥64	≥64	≥64	≥64	≥64	≥64	≥64	≥64	≥64	0
Cefepime	≥64	≥64	≥64	≥64	≥64	≥64	≥64	≥64	32	0
Cefotetan	≥64	≥64	≥64	≥64	≥64	≥64	≥64	≥64	≥64	0
Piperacillin/tazobactam	≥128	≥128	≥128	≥128	≥128	≥128	≥128	≥128	≥128	0
Imipenem (E-test strip)	8	>32	>32	3	32	3	24	4	8	0
Meropenem (E-test strip)	>32	>32	>32	4	16	6	>32	>32	>32	0

Kpn, Klebsiella pneumoniae; Ecl, Enterobacter cloacae; Eco, Escherichia coli; Eae, Enterobacter aerogenes.
